# Automatic Prediction of Recurrence of Major Cardiovascular Events: A Text Mining Study Using Chest X-Ray Reports

**DOI:** 10.1155/2021/6663884

**Published:** 2021-07-09

**Authors:** Ayoub Bagheri, T. Katrien J. Groenhof, Folkert W. Asselbergs, Saskia Haitjema, Michiel L. Bots, Wouter B. Veldhuis, Pim A. de Jong, Daniel L. Oberski

**Affiliations:** ^1^Department of Methodology and Statistics, Faculty of Social Sciences, Utrecht University, Utrecht, Netherlands; ^2^Julius Center for Health Sciences and Primary Care, University Medical Center Utrecht, Utrecht, Netherlands; ^3^Department of Cardiology, Division Heart and Lungs, University Medical Center Utrecht, Utrecht, Netherlands; ^4^Institute of Cardiovascular Science, Faculty of Population Health Sciences, University College London, London, UK; ^5^Health Data Research UK, Institute of Health Informatics, University College London, London, UK; ^6^Central Diagnostic Laboratory, University Medical Center Utrecht, Utrecht, Netherlands; ^7^Department of Radiology, Division of Imaging and Oncology, University Medical Center Utrecht, Utrecht, Netherlands

## Abstract

**Methods:**

We used EHR data of patients included in the Second Manifestations of ARTerial disease (SMART) study. We propose a deep learning-based multimodal architecture for our text mining pipeline that integrates neural text representation with preprocessed clinical predictors for the prediction of recurrence of major cardiovascular events in cardiovascular patients. Text preprocessing, including cleaning and stemming, was first applied to filter out the unwanted texts from X-ray radiology reports. Thereafter, text representation methods were used to numerically represent unstructured radiology reports with vectors. Subsequently, these text representation methods were added to prediction models to assess their clinical relevance. In this step, we applied logistic regression, support vector machine (SVM), multilayer perceptron neural network, convolutional neural network, long short-term memory (LSTM), and bidirectional LSTM deep neural network (BiLSTM).

**Results:**

We performed various experiments to evaluate the added value of the text in the prediction of major cardiovascular events. The two main scenarios were the integration of radiology reports (1) with classical clinical predictors and (2) with only age and sex in the case of unavailable clinical predictors. In total, data of 5603 patients were used with 5-fold cross-validation to train the models. In the first scenario, the multimodal BiLSTM (MI-BiLSTM) model achieved an area under the curve (AUC) of 84.7%, misclassification rate of 14.3%, and F1 score of 83.8%. In this scenario, the SVM model, trained on clinical variables and bag-of-words representation, achieved the lowest misclassification rate of 12.2%. In the case of unavailable clinical predictors, the MI-BiLSTM model trained on radiology reports and demographic (age and sex) variables reached an AUC, F1 score, and misclassification rate of 74.5%, 70.8%, and 20.4%, respectively.

**Conclusions:**

Using the case study of routine care chest X-ray radiology reports, we demonstrated the clinical relevance of integrating text features and classical predictors in our text mining pipeline for cardiovascular risk prediction. The MI-BiLSTM model with word embedding representation appeared to have a desirable performance when trained on text data integrated with the clinical variables from the SMART study. Our results mined from chest X-ray reports showed that models using text data in addition to laboratory values outperform those using only known clinical predictors.

## 1. Introduction

Electronic health records (EHRs) data have become increasingly available to researchers as more hospitals, clinics, and practices have adopted data digitization. EHRs store data in different modalities, such as structured data (e.g., demographic values, laboratory results, and medications) and unstructured texts (e.g., referral letters, clinical notes, discharge summaries, and radiology reports). This digitization creates an opportunity to mine the health records to increase the quality of care and clinical outcomes. Yet, clinicians have limited time to process all the available data and detect patterns across similar medical records. Deep learning and machine learning, on the other hand, are suitable for discovering useful patterns from a vast amount of data.

Unstructured texts contained within the EHRs are recognized as a rich but not easily accessible and usable source of medical information [1–6]. Recent studies have attempted to derive information from unstructured medical texts to classify disease codes [7–10], detect patient's disease history [11, 12], and predict hospital readmission or clinical outcomes [13–15]. X-ray radiology reports are an example of such unstructured data describing radiologist's observations on patient's medical conditions associated with medical images. The majority of previous decision support systems for radiology reports are developed using rule-based approaches applied on unstructured and semistructured texts [16–19]. However, these methods are often impractical because they do not generalize to new data and often are not applicable for big data analysis [20].

Recent studies have shown promising results using free-text radiology reports and deep learning models to predict clinical outcomes [17, 21–25]. Convolutional neural networks (CNNs) and recurrent neural networks (RNNs) are two common deep learning techniques that have been effective in text mining and natural language processing (NLP), as well as EHR applications [7, 15, 21, 26, 27]. Deep learning-based modelling of radiology reports has been proposed to supersede the simple grammatical patterns and hand-crafted regular expressions of the traditional clinical rule-based software, such as PEFinder [28], MedLEE [29, 30], and CTakes [31]. While these neural networks models gained tremendous momentum in knowledge discovery from EHR texts, there are very seldom studies that used both free-texts and structured information in EHRs for clinical prediction and classification [32–35].

In this paper, we leveraged structured features in EHR data to combine with free-text radiology reports to uncover patterns to improve cardiovascular risk prediction. Free-text within EHRs might contain additional information for clinical prediction modelling, either as an added variable to improve prediction performance compared to current models or as an auxiliary variable to increase the flexibility of prediction in the case of inaccessible clinical data.

The contributions of this study are twofold. The first contribution is to develop and evaluate a text mining pipeline for capturing additional information from text. The second is the use of chest X-ray reports from routine care as free-text in combination with the laboratory values, collected in the Second Manifestations of ARTerial disease (SMART) study [36], in a multimodal architecture to predict the recurrence of cardiovascular events in cardiovascular patients.

## 2. Materials and Methods

In this section, we describe the case study, data ethics and privacy, and the details of our proposed text mining pipeline.

### 2.1. Case Study

#### 2.1.1. Patient Population

The patients included in this study were originally included in the SMART  study. The  design of the SMART study is published elsewhere [36]. In short, the SMART study is an ongoing single-center prospective cohort study designed to establish the presence of additional arterial disease and risk factors for atherosclerosis in patients with vascular disease or a vascular risk factor. Patients visiting the University Medical Center (UMC) Utrecht for evaluation of any atherosclerotic cardiovascular condition are eligible for inclusion in SMART. The inclusion criteria are presenting with an atherosclerotic cardiovascular condition and age >18 years. Exclusion criteria are life expectancy <3 months, unstable vascular disease, and insufficient fluency in the Dutch language. A total of 5603 SMART  patients were included in this analysis. The characteristics of the patients are listed in Table 1.

#### 2.1.2. Clinical Variables

Variables that are predictors in the SMART  study [36] (age; sex; smoker; systolic blood pressure; diabetes; HDL cholesterol; total cholesterol; renal function according to the MDRD formula; history of cardiovascular disease stratified for stroke, peripheral artery disease, abdominal aortic aneurysm, and coronary heart disease; and years since diagnosis of first cardiovascular disease) were used for prediction modelling for all patients.

#### 2.1.3. Chest X-Ray Reports

Free-text reports from chest X-rays that were taken in SMART  patients, which were made in routine care, were extracted from their EHR and included in this analysis.

#### 2.1.4. Ethics and Privacy

Informed consent was obtained through established procedures. The SMART study was approved by the Medical Ethical Committee of the UMC Utrecht. All data are handled according to local data protection guidelines and privacy regulations.

### 2.2. Text Mining Pipeline

Figure 1 illustrates the text mining pipeline for the prediction task. The goal  is to forecast the major cardiovascular events (MACE) during follow-up as the outcome prior to clinical variables and chest X-ray reports.

#### 2.2.1. Preprocessing

Clinical variables were preprocessed by missing value imputation and a normalization step. Missingness of data was solved using the MICE package [37] with one imputation for each missing value. As an additional normalization step, the clinical variables were rescaled to homogenize their levels of variance.

In preprocessing the radiology reports, the following steps were performed to improve the quality of text data for the subsequent steps: (1) all characters were transformed into lowercase; (2) we removed numbers and some meaningless punctuation marks, such as semicolons and colons; and (3) stop words were then removed. Dutch stop words used in this study are shown in Table 2. (4) We then applied Porter's stemming algorithm [38, 39] to texts.  Figure 2 shows the 20 most frequent words before and after the preprocessing step for the X-ray radiology report in the SMART study. “Klinisch (clinical)” and “xthorax (chest X-ray)” appeared in all reports as they denote the indication of the test and type of X-ray; therefore, we removed them as noninformative stop words. Other words were merged into their stem words.

#### 2.2.2. Representation and Feature Extraction

Text representation includes dimensions in which text is represented in a vector space model. We explored three text representation techniques used in the text mining pipeline:

- Bag-of-words (BOW)
- Clustering-based representation
- Word embedding

We used three different techniques: an interpretable method, a method with a low-dimensional output, and a less interpretable and more semantic-based technique to be able to assess their differences in performance in mining additional information for clinical prediction modelling.

*(i) Bag-of-Words*. The BOW representation is the most commonly used representation for text mining applications [11]. Words in the reports were converted into a sparse multidimensional representation, which was leveraged for further classification and clustering purposes. Representation of text includes frequencies of words per patient's text report. This is a method that is relatively easy to understand and interpret for clinicians.

*(ii) Clustering-Based Representation*. We applied latent Dirichlet allocation (LDA) [40] to further cluster the BOW representation of patient radiology reports. LDA is a topic modelling approach that groups a collection of documents to obtain the probabilities of the distributions of document–topic and topic–word in the data set. This method has the advantage of using an interpretable lower-dimensional representation of text and the disadvantage of lacking the capacity of methods that use all features of unstructured medical notes. We ran the experiments fitting the LDA topic model with Gibbs sampling [11, 40] using 10 topics.  Figure 3 shows two topics of the output of LDA applied to the X-ray radiology reports in the SMART study. Potential clinical scenarios that fit these topics are (a) possible cardiac decompensation and (b) possible pneumonia.

*(iii) Word Embedding*. Neural network-based word embedding incorporates not only the contexts of a word but also the semantic relation with other words [1, 41, 42]. We used a window of five words for the context words that were used in this representation technique. Subsequently, word vectors were aggregated for each patient report.

#### 2.2.3. Classification Algorithms

In the text mining pipeline, independent variables are the clinical variables and features extracted from radiology reports, though these features differ per text representation approach. MACE as defined by the SMART study was used as an outcome variable. We made a total of six different algorithms to be able to study both baseline and the state-of-the-art machine learning methods and their additional value for clinical risk prediction.

*(i) Baseline Models*. Using traditional machine learning classifiers, we applied an LR model and a support vector machine (SVM) algorithm to data from the SMART case study. If the interpretation of a model is of primary interest, LR parameters can easily be interpreted in terms of the log odds. SVM on the other hand is a supervised learning technique that produces nonlinear boundaries by constructing a linear boundary in a large, transformed version of the feature space, and it scales relatively well to high dimensional data, such as unstructured texts [43].

*(ii) Deep Learning Models*. We studied using the state-of-the-art deep learning methods: a CNN, a long short-term memory (LSTM) RNN, and a bidirectional LSTM (BiLSTM) [7, 15, 21, 26]. We also employed a feed-forward multilayer perceptron neural network for the case of no text presented to the model. However, multilayer perceptron is not well adapted to textual data [1, 8, 26]. This is because it is defined for vectors as input data; hence, to apply it to texts, we must transform the texts into vectors. CNN, LSTM, and BiLSTM are deep learning architectures that have removed the manual extraction of features from text data.

#### 2.2.4. Multimodal Neural Network

Figure 4 illustrates the proposed deep learning-based architecture for the text mining pipeline. In this architecture, we propose a multimodal learning model using a BiLSTM deep neural network.

The multimodal neural network architecture consists of an embedding layer, a BiLSTM layer, a dropout, a concatenation layer, and dense layers.

#### 2.2.5. Embedding Layer

To extract the semantic information of radiology reports, each text is firstly represented as a sequence of word embeddings. Word embedding is an improvement over the bag-of-words models where large sparse vectors were used to represent each word. On the contrary, in an embedding, words are represented by dense vectors where a vector represents the projection of the word into a continuous vector space [41, 42]. Denote *s* as an X-ray report with *m* words and each word is mapping to a vector; then, we have

(1) $$\begin{array}{c} s=\left[{\overset{⟶}{e}}_{1},{\overset{⟶}{e}}_{2},\ldots ,{\overset{⟶}{e}}_{m}\right], \end{array}$$

where vector ${\overset{⟶}{e}}_{i}$ represents the vector of *i*-th word with a dimension of *d*. The  vectors of word embeddings are concatenated together to maintain the order of words in a patient report.

#### 2.2.6. Bidirectional-LSTM Layer

After the embedding layer, the sequence of word vectors is fed into a bidirectional LSTM layer to achieve another representation of radiology reports. Interest in incorporating a BiLSTM layer into the architecture of our model arises from their ability to learn long-term dependencies and contextual features from both past and future states [44]. The BiLSTM layer calculates two parallel LSTM layers, a forward hidden layer, and a backward hidden layer, to generate an output sequence *y* as illustrated:

(2) $$\begin{array}{c} h_{f_{t}}=\sigma \left(W_{xh_{f}}x_{t}+W_{h_{f}h_{f}}h_{f_{t-1}}+b_{h_{f}}\right),\\ h_{b_{t}}=\sigma \left(W_{xh_{b}}x_{t}+W_{h_{b}h_{b}}h_{b_{t-1}}+b_{h_{b}}\right),\\ y_{t}=W_{h_{f}y}h_{f_{t}}+W_{h_{b}y}h_{b_{t}}+b_{y}, \end{array}$$

where *σ* is the sigmoid activation function; *xt* is a *d*-dimensional input vector at time step *t*; *W* are the weight matrices; *b* are bias vectors; and *h*_*f*_ and *h*_*b*_ are the output of the LSTM forward and backward layers, respectively.

The multimodal BiLSTM integrates the neural text representation with clinical predictors and feeds them into a fully connected neural network. We used a BiLSTM network to connect both previous and future information to the present information in text reports. This was made possible by having two propagating networks in opposite directions: one network running from the beginning of the text to the end and the other in the opposite direction. These forward and backward networks memorize information about the report from both directions. Thus, the context window around each word consists of information both prior to and after the current word. In this way, BiLSTM can model the entire sequence of words in a radiology report to capture dependencies between the feature space and the relationship with the outcome variable.

#### 2.2.7. Other Deep Neural Networks

When applying a CNN model to our architecture, we used a convolution layer with a max pooling layer instead of the BiLSTM layer in the architecture in Figure 4. For employing an LSTM model, only the left to the right direction in the text is monitored inside the hidden RNN layer.

### 2.3. Evaluation Measures

To evaluate the classification performance of our text mining pipeline, we used five available metrics: area under the curve (AUC), misclassification rate, precision (positive predictive value), recall (sensitivity), and F1 score. AUC is the area under the receiver operating characteristic curve, which is created by plotting the true positive rate against the false positive rate. Misclassification rate is the proportion of incorrectly classified instances made by a model. Precision is the fraction of relevant instances among the retrieved instances, while recall is the fraction of relevant instances that have been retrieved over the total amount of relevant instances. The F1 score can be interpreted as a weighted average of precision and recall. The relative contributions of precision and recall to the F1 score are equal. The formulae of precision, recall, and the F1 score are defined in the following:

(3) $$\begin{array}{c} \text{precision}=\frac{\text{true positive}}{\text{true positive}+\text{false positive}},\\ \text{recall}=\frac{\text{true positive}}{\text{true positive}+\text{false negative}},\\ \text{F}1\text{ score}=\frac{2*\text{precision}*\text{recall}}{\text{precision}+\text{recall}}. \end{array}$$

## 3. Results

Our pipeline was implemented in *Python* and *R* using various text mining, NLP, and machine learning packages. The multimodal learning architecture was implemented on *Keras* with a *TensorFlow* backend (https://keras.io). The source code is publicly available at GitHub (https://github.com/bagheria/CardioRisk-TextMining). We performed 5-fold cross-validation for all experimental analyses. We used the hyperparameter setting as shown in Table 3. These hyperparameters were tuned based on the validation set. We used the embeddings with a vector size equal to 500 and a window size equal to 5. In addition, we set the number of filters in the CNN to 128 and the filter size to 5. The hidden dense layers contained 64 units and used the *ReLU* activation function, and the output layer used a *sigmoid* activation function. We set the same number of hidden units in the LSTM layers at 100. Both dropout and recurrent dropout were added at 0.2 to avoid overfitting [45]. We set the batch size and number of epochs to 64 and 20, respectively.

To assess the added value of text for the prediction of MACE, we compared various scenarios of clinical variables and text reports in the proposed text mining pipeline:

1. Prediction using only radiology reports (models starting with T)
2. Prediction using only clinical variables (models starting with V)
3. Prediction using the integration of clinical variables and radiology reports (models starting with VB, VC, and MI)
4. Prediction using only sex and age variables (models starting with D)
5. Prediction using the integration of sex and age variables and radiology reports (models starting with DB, DC, and D-MI)

Table 4 lists the experimental results for AUC and the misclassification rate for the first three scenarios. In these experiments, we evaluated different models using only clinical variables, only radiology reports, and their integration.

V-LR, V-SVM, and V-NN are the models trained on only clinical variables. The features in these models included the SMART variables as independent variables and MACE during follow-up as the outcome in prediction models. T-SVM, T-LR, and T-BiLSTM are the models with only text reports as their predictors. T-SVM was trained on the BOW representation of the reports. T-LR used the clustering-based representation. In this scenario, we reported each model's best result among representation methods. T-SVM achieved the highest performance in this scenario with an AUC of 62.5% and a misclassification rate of 18.6%. VB and VC are the models trained on clinical variables combined with the BOW and clustering-based representations, respectively. VC-SVM gained the lowest AUC of 65.5%, while the VB-SVM model obtained the lowest misclassification rate of 12.2%.

MI represents the models that used the proposed multimodal learning architecture with the neural word embedding representation. In this scenario, MI-BiLSTM, MI-LSTM, and MI-LR achieved promising results. MI-BiLSTM obtained the highest AUC of 84.7% and the lowest misclassification rate of 14.3% in this case. MI-LR still has the second ranking AUC at 81.1%.

Precision, recall, and F1 score evaluation measures are recommended for imbalanced data, where the AUC and misclassification rate may provide an optimistic view of the performance [46].  Figure 5 shows the performance of the models using precision, recall, and F1 score metrics. The deep learning models achieved better performance compared to other models in different scenarios. The MI-BiLSTM model achieved the highest performance in terms of all evaluation measures. The F1 score was 83.8%. MI-LSTM and MI-CNN obtained F1 score performances of 78.9% and 74.7%, respectively. These results are evidence of the performance of text mining techniques with multimodal learning architecture in extracting knowledge from radiology reports and combining them with classical clinical predictors. It is notable that the multilayer perceptron neural network achieved promising results when trained only on clinical variables. This model obtained a precision of 75.1%, recall of 79.4, and F1 score of 77.2%. This shows the efficiency of the neural network model and the relatedness of the laboratory results in predicting cardiovascular risk.

To assess the value of text as additional variables if clinical predictors are not available, we again compared the abovementioned scenarios but with only sex and age as clinical variables.  Table 5 lists the results of this evaluation of the text mining pipeline. We named the models in this scenario D-models to show that they have been trained on demographic (age and sex) features.

The D-MI-BiLSTM model gained the highest AUC of 74.5%. D-MI-BiLSTM was trained using the multimodal architecture, meaning that it used the neural word embedding representation and BiLSTM hidden layer output to concatenate the radiology reports with age and sex. DB-SVM gained the lowest misclassification rate of 16.3%. This model was trained on the combination of the BOW representation and the age and sex variables.

In Figure 6, the results of precision, recall, and F1 score are compared for the scenarios when clinical predictors are not available. This setting also confirms that text mining-based models achieved better performance when predicting the MACE variable. The D-MI-BiLSTM, D-MI-LSTM, and D-MI-CNN models gained F1 scores of 70.8%, 67%, and 64.3%, respectively. The LR model with only age and sex only reached 44.2%, 49.4%, and 46.66%, respectively.

## 4. Discussion

This study aimed to develop and evaluate a text mining pipeline integrating clinical and text variables applied to cardiovascular risk prediction. Our research (1) integrates EHR structured laboratory results and unstructured radiology text in a text mining pipeline to make an accurate decision for classifying cardiovascular events; (2) uses routine care data including X-ray reports in Dutch for cardiovascular risk prediction; and (3) incorporates free-text reports as auxiliary variables when classical predictors are not available. In our experiments for the SMART case study, we found that neural text representation and prediction modelling significantly add to baseline models with classical clinical predictors to predict MACE. In the case of unavailable clinical predictors, the proposed MI-BiLSTM model with just age, sex, and word embedding attains a similar discriminative performance to that of the models trained on the classical SMART variables. Deep learning methods are increasingly being adopted in the medical field. For example, in radiology, deep learning has shown remarkable results in image analysis [47], and in intensive care, RNNs have been used to determine variables that are proxies for clinician decision-making [48]. The application of text mining and NLP in the predictive setting is not new; unlocking the full potential of EHR data is contingent on the development of text mining pipelines to automatically transform free-text into structured clinical data that can guide clinical decisions [1, 2, 4, 49]. Yet, text as auxiliary variables to classical clinical variables has only been considered in a few studies [32–34, 50, 51]. One study [51] predicted several clinical interventions combining structured data and clinical notes. Each clinical narrative note was transformed to a 50-dimensional vector of topic proportions for each note using an LDA algorithm. This resulted in a lower-dimensional representation of text, losing the depth of information in unstructured text. Another study [33] extracted structured information from clinical notes using regular expression and a heuristic rule-based tool. Again, this is a method that uses a general framework for predicting the onset of diseases, combining both free-text medical notes and structured information. The mined text was then used to predict congestive heart failure, kidney failure, and stroke via deep learning models, achieving good performance in disease prediction. Lastly, one study [34] combined unstructured text, semistructured text, and structured data in machine learning models. Separate models were developed to handle data from different modalities to create an ensemble model that predicts diagnostic codes of the international classification of diseases (ICD-10). Hence, in this study, we combine all advantages of prior research by developing a machine learning-based modelling of radiological language, to integrate clinical variables and textual features, to supersede traditional algorithms using only clinical variables. In this paper, we explained how we used text preprocessing techniques and applied text representation methods to chest X-ray reports. These representations were then used as auxiliary variables to the clinical variables from the SMART study to predict MACE using six different classification techniques.

There are strengths and limitations to our case study. Because patients must have had an indication for a routine care chest X-ray, there was a selection in the case study. However, this does not in fact mean there is selection bias; it merely restricts the generalizability of the clinical prediction model to cardiovascular patients without an X-ray report available. Pragmatically, we hypothesize that using available information–including bodies of text, such as this chest X-ray report–for predictions rather than a strict set of predictors will make predictions more flexible and more tailored to individuals. The use of advanced techniques, such as text mining, in clinical practice requires support for implementation. Implementation includes the application of the mining pipeline and integration in the care process using technologies, such as computerized decision support (CDSS). CDSS allows technical results from algorithms, such as text mining, to be translated to practical suggestions for clinical practice. To help clinicians interpret results that come from text mining, collaborations between technical text mining experts (biostatisticians, mathematicians, data scientists, and software engineers) and practical experts (clinicians) are needed to safeguard the technical quality and medical relevance. Future studies will focus on two points. First, our multimodal learning architecture will be validated for other similar scenarios, such as adverse event monitoring, hospital readmission, or disease classification, in which both EHR structured variables and free-text reports would contribute to the judgement of final outcomes. Secondly, we will expand our pipeline to a model to use the available clinical dictionaries with machine learning and deep learning models. The publicly available source code of our model (https://github.com/bagheria/CardioRisk-TextMining) can be used to evaluate performance on potentially clinically relevant classification tasks based on clinical notes and EHR variables.

## 5. Conclusions

Medical free-text potentially contains valuable information for clinical decision-making. Text mining methods are the key to the successful extraction of clinically important findings from these free-text reports. Medical text mining is a step-by-step process that requires tailoring to the aim of the project and the context of reports. Text mining potentially opens the door to valuable information captured in free-text medical data. We believe that such models are useful in reducing work overload for clinicians by providing the needed clinical decision support.

## Figures and Tables

**Figure 1:** Methodology text mining pipeline overview.

**Figure 2:** Most frequent words in the X-ray radiology reports in the SMART  study. (a) Initial top frequent words. (b) Top frequent words after preprocessing.

**Figure 3:** LDA clustering. The *y*-axis shows the top words in the selected cluster (topic). The *x*-axis shows the probability of the word in the topic. (a) Possible cardiac decompensation. (b) Possible pneumonia.

**Figure 4:** Proposed multimodal learning architecture with a deep learning model.

**Figure 5:** Comparison of precision, recall, and F1 score for experimental scenarios.

**Figure 6:** Comparison of precision, recall, and F1 score for experimental scenarios when clinical predictors are not available.

**Table 1:** Characteristics of the patients.

Characteristics	Total *n* = 5603
Age, years, mean (SD)	56.2 (12.5)
Female sex, *n* (%)	1926 (34.4)
Current smoker, *n* (%)	1549 (27.6)

*History of*CVD	
CHD, *n* (%)	2166 (38.7)
Stroke, *n* (%)	1076 (19.2)
PAD, *n* (%)	631 (11.3)
AAA, *n* (%)	306 (5.5)
Years since first diagnosis of CVD, median (IQR)	0 (0–4)

*Risk factors for CVD*	
Diabetes mellitus, *n* (%)	1047 (18.7)
Hypertension, *n* (%)	2353 (42.0)
Dyslipidemia, *n* (%)	432 (7.7)
BMI, kg/m^2^ (mean (SD))	26.8 (4.3)
SBP, mmHg (mean (SD))	140 (21)
DBP, mmHg (mean (SD))	83 (13)
Total cholesterol, mmol/L (mean (SD))	5.14 (1.38)
LDL-cholesterol, mmol/L (mean (SD))	3.1 (1.16)
HDL-cholesterol, mmol/L (mean (SD)	1.27 (0.38)
Triglycerides, mmol/L (median (IQR))	1.7 (1.2–2.5)
MDRD, ml/min/1.73 m^2^ (median (IQR))	80 (68–91)
HbA1*c*, mmol/mol (median (IQR))	5.7 (5.4–6.1)
Glucose, mmol/L (median (IQR))	5.7 (2.6–6.4)
Hemoglobin, mmol/L (mean (SD))	6.0 (2.04)
Creatinine, *μ*mol/L (median (IQR))	84 (73–97)
CRP, mg/L (median (IQR))	1.95 (0.90–4.20)
TSH, mU/l (mean (SD))	0.9 (0.09)
MACE during follow-up, *n* (%)	1385 (24.7)

CVD: cardiovascular disease; CHD: coronary heart disease; PAD: peripheral arterial disease; AAA: abdominal aortic aneurysm; BMI: body mass index; SBP: systolic blood pressure; DBP: diastolic blood pressure; LDL: low-density lipoprotein; HDL: high-density lipoprotein; MDRD: modification of diet in renal disease; HbA1c: hemoglobin; A1c CRP: C-reactive protein; TSH: thyroid-stimulating hormone; MACE: major cardiovascular events.

**Table 2:** Dutch stop words used in this case study.

de	informatie	je	al	na	worden	tegen
en	eerdere	mij	waren	reeds	zelf	gegevens
van	klinisch	uit	doen	wil	ons	klinische
ik	er	der	toen	kon	kunnen	tot
te	maar	daar	moet	uw	ook	omdat
dat	om	haar	ben	iemand	bij	ge
die	hem	naar	kan	geweest	zich	nu
in	dan	heb	hun	andere	gegevens	had
aan	zou	hoe	dus	klinisch	voor	als
een	of	heeft	onder	informatie	hier	thorax
hij	wat	hebben	ja	gegeven	men	u
het	mijn	deze	eens	xthorax	zijn	doch
is	dit	want	wie	conclusie	met	me
was	zo	nog	werd	onderzoek	ze	zij
op	door	zal	altijd	opname	wordt	eerder
over	ter	x/x				

**Table 3:** Hyperparameter setting.

Hyperparameter	Value
Embedding size	500
Window size	5
#filters	128
Filter size	5
#hidden units	64
Hidden activation function	ReLU
Output activation function	Sigmoid
#LSTM units	100
Dropout	0.2
Recurrent dropout	0.2
Batch size	64
#epochs	20

**Table 4:** Performance comparison of different experimental scenarios using AUC and misclassification rate.

Classifier	AUC	Misclassification rate
V-LR	0.799	0.195
V-SVM	0.648	0.196
V-NN	0.651	0.201
T-LR	0.512	0.247
T-SVM	0.625	0.186
T-BiLSTM	0.570	0.300
VB-LR	0.808	0.193
VB-SVM	0.784	0.122
VC-LR	0.809	0.194
VC-SVM	0.655	0.197
MI-LR	0.811	0.203
MI-SVM	0.694	0.237
MI-CNN	0.730	0.214
MI-LSTM	0.794	0.176
MI-BiLSTM	0.847	0.143

**Table 5:** Performance comparison of different experimental scenarios using AUC and misclassification rate when clinical predictors are not available.

Classifier	AUC	Misclassification rate
D-LR^*a*^	0.685	0.242
D-SVM	0.572	0.246
D-NN	0.567	0.214
DB-LR^*b*^	0.703	0.247
DB-SVM	0.674	0.163
DC-LR^*c*^	0.705	0.239
DC-SVM	0.534	0.247
D-MI-LR^*d*^	0.708	0.235
D-MI-SVM	0.568	0.247
D-MI-CNN	0.667	0.228
D-MI-LSTM	0.708	0.209
D-MI-BiLSTM	0.745	0.204

^*a*^LR trained on demographic variables. ^*b*^LR trained on demographic variables and BOW representation. ^*c*^LR trained on demographic variables and clustering-based representation. ^*d*^Multimodal learning LR trained on demographic variables and word embeddings.

## Data Availability

The dataset is not publicly available due to patient privacy restrictions.
